# Situation and Countermeasures of the Management Team of the Elderly Care Institutions from the Perspective of the Combination of Medical and Health Care: A Cross-Sectional Study

**DOI:** 10.1155/2020/8826007

**Published:** 2020-09-02

**Authors:** Li Yang, Hongmei Peng, Yunfan Yang, Linqi Ouyang, Yunfeng Li

**Affiliations:** ^1^Science and Technology Department, Changde Vocational Technical College, Changde, Hunan 415000, China; ^2^Scientific Research and Education Department, The First People's Hospital of Changde City, Changde, Hunan 415000, China; ^3^Scientific Research Department, Changde Federation of Social Sciences, Changde, Hunan 415000, China

## Abstract

**Objective:**

In order to provide evidence for improving the quality of managers in elderly care institutions, this paper explored the situation of managers of elderly care institutions in a city in Central China under the national guidelines for the combination of medical and elderly health care.

**Design:**

A cross-sectional study carried out in a city in Central China was designed. *Setting*. The online questionnaire was distributed to the managers of six elderly care institutions in a city in Central China. *Participants*. The questionnaire was sent to 61 recipients; from this, 60 responses were obtained.

**Results:**

There was a 98% response rate. The study found that most managers in elderly care institutions were middle-aged, with low education level and years of management. The job mobility was high, and 27% of the managers had no relevant certificates. Management years had a significant influence on the rate of certificate holding (*P* < 0.05). Some managers were less than 30 years old and had college degree or above, which indicated that people with young and high levels of education were more likely to become managers. However, there was no significant difference in educational level among managers of different ages (*P* > 0.05). 56.6% of the managers have received provincial or municipal training, and few managers have received the national level training. The education level is positively related to the access to training opportunities. More than half of the managers earn less than ¥3000 a month. The study showed that the education level was positively related to the career growth space (*P* < 0.05).

**Conclusions:**

Specialized training and high salary should be provided for managers to improve their elderly care skills and hence the quality of elderly care service. In addition, in order to improve the education level of managers, a long-term continuing education system should be established gradually. Through expanding the enrollment scale of the nursing school, carrying out training about elderly care skills, and issuing vocational skills certificates to those who pass the examination, the number of local nurses for the elderly will be increasing, and the quality of the elderly care service will be improving.

## 1. Introduction

According to the law of the People's Republic of China on the protection of the rights and interests of the elderly, the elderly refers to citizens over the age of 60. According to the international classification standard, the aging country refers to a country or region where the proportion of the population aged 60 and above in the total population exceeds 10% or the proportion of the population aged 65 and above in the total population exceeds 7%. A study shows that China has already entered an aging society, and the aging process is accelerating. The number of the elderly over 80 years old is increasing at the rate of 1 million per year [1]. At the end of 2016, there were 230.86 million people aged 60 and over in China, accounting for 16.7% of the total population, and 15.03 million people aged 65 and over [2]. By 2020, there will be 248 million people aged 60 and over in China, and by 2050, there will be more than 318 million people, accounting for more than 30% of the total population. China will enter into a society of severe aging and become the country with the largest elderly population in the world. Among the permanent residents of a city in Central China, 21.3% are over 60 years old and 14.7% are over 65 years old, and the elderly population is growing.

The problem of aging in China is becoming more and more serious, and the problem of providing elderly care has become a hot topic. There is a concept that there is a large demand for elderly care, but the service quality of the elderly care is low [3]. Sweden has formulated the health and medical service law, which emphasizes that it is the right of every citizen serviced on medical care [4]. The United States adopts a long-term care model that combines voluntary and compulsory care, among which the representative is pace plan and long-term care insurance (LTC). The combination of medical and health care refers to the combination of medical resources and elderly services resources, which is the integration of medical treatment, rehabilitation, health preservation, and elderly care. Its biggest feature is not only to provide clinical diagnosis and treatment for the elderly but also to provide life care, physical rehabilitation, and hospice care. In addition, the combination of medical care and health care not only provides traditional day care, entertainment, mental support, and other services but also provides the elderly with disease treatment, rehabilitation, regular physical examination, hospice care, and other services [5].

The national guidance on accelerating the development of the elderly care service industry issued by the State Council in 2013 proposed that the development of the combination of medical care and elderly care should be promoted, and a new mode of cooperation between medical institutions and elderly care institutions should be explored [6].

In November 2015, the Health and Family Planning Commission and the Ministry of Civil Affairs and other departments issued the guidance on promoting the combination of medical and elderly care services, emphasizing the integration of medical treatment and elderly care. In 2016, the General Office of the State Council put forward the guidance on exploring a quick way for the development of the combination of medical care and health care, and establishing medical and health institutions such as geriatric hospitals, rehabilitation hospitals, infirmaries, and so on. In addition, the guidance pointed out that the qualified elderly care institutions should be included in the designated scope of urban and rural basic medical insurance [7].

In April 2019, the Document No. 5 about promoting the development of elderly care service issued by the General Office of the State Council, or guidance for short [8], reported that it was essential to improve the ability of combining medical and health care services, with expanding employment and entrepreneurship of elderly care services. According to the guidance of Department of Aging Health of National Health Committee on further promoting the development of the combination of medical and health care in Document No. 60 in 2019, the reforms to streamline administration and delegate power, ease restrictions, and strengthen regulation where necessary, and improved services for the integration of medical and health care should be promoted [9]. Meanwhile, nongovernmental sectors running medical and elderly care institutions should be encouraged. Meanwhile, local governments should be encouraged to formulate various preferential policies to support these institutions according to the local conditions.

### 1.1. Design and Setting

The data used in this study were from a cross-sectional survey conducted at six elderly care institutions in a city in Central China. A questionnaire survey was conducted among the managers of six elderly care institutions in the city, and 1-2 principals of each institution were interviewed in depth. With the consent of the leads of the local Civil Affairs Bureau and the relevant departments of the Aging Committee, the research team contacted the leads of the elderly care institutions for support.

In the first stage, the researchers accepted formulated standards and training of survey to understand the purpose, methods, and contents of the study. Then, the research team conducted questionnaire survey and interview to explain the purpose and significance of the research to managers of the institutions in detail. The questionnaire was filled in one-to-one way, and the researchers explained the contents of the filled items in detail. The questionnaire was completed by trained researchers, and the questionnaire was entered by the double entry method to ensure the accuracy of the data. In the second stage, the interview contents of the principals of the institution include the elderly care service mode, character of the institution, establishment of the institution and department, allocation and area of the health care room, number and setting of beds, total number and positions of the staff, number and distribution of the managers, number of the doctors and nurses, number of social workers, training arrangement of the staff, combination of medical and health care service project, and measures adopted for the stability of the management team. In the third stage, The interview contents for managers include the basic information, age, education level, specialty (nurses, doctors, social workers, and volunteers), salary, professional certificate, working years, daily working hours, working contents, previous work, relevant training received, willingness to engage in elderly care service, and measures to improve the welfare of managers in elderly care institutions.

The questionnaire based on the national guidelines and literature review for elderly care offered to managers of elderly care institutions was sent electronically to the managers. The self-made questionnaire involved 18 items, which were the age, gender, household registration, education level, management years, qualification, postadaptation, sleep status, job burnout, professional affection, career development space, monthly income, expected monthly salary, career prospect, job mobility, training situation, and desired training situation. Professional affection included professional identity, sense of honor, job satisfaction, and empathy.

### 1.2. Statistical Analysis

The original data were input by Excel, and SPSS18.0 software was used for descriptive analysis of data, which were expressed by composition ratio, rate, frequency, and percentage. Fisher's exact test was used to explore the possible factors related to the management years, education level, career growth space, income, and training opportunity.

## 2. Results

### 2.1. Professional Characteristics of Managers

A total of 61 questionnaires were distributed to all elderly care institutions in a city in Central China. From these, 60 questionnaires were fully completed and returned. They were 20 males and 40 females, and their average age is 40.81 ± 4.32. Among these, managers, presidents, vice presidents, and chairmen in different elderly care institutions were 7. 18 managers in the nursing department, 10 personnel in the human resources department, and 25 others were included. 70% participants were residences of the city.

The ratio of men and women in the management of the elderly care institutions was 1 : 2, which indicated that women were more willing to engage in elderly care services. The average age of managers was 40.81 ± 4.32 years old, and 45% of them were 40–50 years old. The education level of managers was low, with 40% of them in middle school or high school and 25% under middle school. 70% of managers were local residents, which was related to the traditional idea that Chinese women at home were family oriented, and they can take good care of their families if they work nearby. The management years of managers were mostly 2–5 years, which showed that the job mobility of managers was relatively large (Table 1).

### 2.2. Managers Have Low Certificate Holding Rate, Less Professional Training, and Lack of Professional Knowledge

Some managers did not have relevant qualifications, accounting for 27%, which indicated that the certificates holding rate is low. The qualifications mainly included the elderly nurse certificate, clinical nurse certificate, and social worker certificate (Table 2). The result showed that management years had a significant influence on the rate of certificate holding (*P* < 0.05). There were 15 managers under middle school, accounting for 25%. Among them, 6 managers aged 51–60, accounting for 35.29%. 40% managers had middle school or high school education. Some managers were less than 30 years old, with college degree or above, which indicated that young and high levels of education were more likely to become managers (Table 3). However, there was no significant difference in the educational level among managers of different ages (*P* > 0.05). The proportion of elderly care-related majors among managers was low. The majority of managers received training in workplace, accounting for 70%. 56.6% of managers have received provincial or municipal training, and few managers have received the national level training. The government provided less training opportunities for these managers, and most of management knowledge comes from their work experience. There were 39 managers who wanted to acquire knowledge and skills of communication through training, 31 managers who wanted to acquire management and marketing knowledge, and 30 managers who wanted to acquire medical and nursing knowledge. The results showed that the lower the education level, the more training in workplace, while the higher the education level, the more opportunities for national and provincial training. The education level was positively related to the training opportunities (Figure 1).

### 2.3. The Job Satisfaction and Salary of Managers Are Low, the Space for Career Growth Is Little, and the Job Burnout Is Strong

Nearly 50% of managers were satisfied with their work, but 15% were still not satisfied with their work status. The main reasons for their dissatisfaction included overwork, fatigue, and low income. 80% of managers felt tired, while less felt ease at work. According to the data of the National Bureau of statistics, in 2018, the annual disposable income of Chinese residents was ¥28228, and that of a city in Central China was ¥24241, ranking 13th in China. In 2019, the annual disposable income of residents in the city was ¥27680, including ¥25101 in Dongting Lake area (Yueyang City, Changde City, and Yiyang City), an increase of 9.5%. In the same year, the annual disposable income of urban residents and rural residents was ¥39842 and ¥15395, respectively. The result showed that the average monthly income of managers was ¥3436, 3.33% of which was lower than ¥2000 and 58.33% of which was ¥2000-3000. More than half of the managers had a monthly income of less than ¥3000, and only one manager had more than ¥5000. The average monthly salary of managers is far lower than the per capita disposable income of urban residents in the city. 20% of managers believed that there was no room for career growth, while 50% felt there was room for growth, but not much. The lower the education level of managers, the smaller the room for them to rise. Managers with bachelor's degree believed that they had a lot of room for career growth. 25% of managers thought it would take time to change their career prospects. The data showed that education level has a significant impact on the career growth space (*P* > 0.05), and managers with the higher education level have a larger career growth space (Table 4). However, there was no significant difference in the salary level of managers with different education levels (*P* > 0.05) (Table 5).

## 3. Discussion

### 3.1. Comprehensive Training of Personnel in Elderly Care Institutions Should Be Provided

The results showed that most managers in elderly care institutions were middle-aged, with low education levels and clinical management years. 25% of managers had a diploma below middle school, and 27% of the managers had no relevant certificates. The rate of certificate holding was low. Few managers have received the national level training. There were 39 managers who wanted to acquire knowledge and skills of communication through training, 31 managers who wanted to acquire management and marketing knowledge, and 30 managers who wanted to acquire medical and nursing knowledge. As of September 2017, the total number of elderly care institutions has exceeded 144600, an increase of 226% compared with 44300 at the end of 2012 [10]. Most of the elderly living in the elderly care institutions are the elderly with chronic disease, semidisability, or disability. Therefore, on the basis of providing daily life care, the elderly care institutions are required to undertake the life care, health management, psychological intervention, nutrition catering, part of medical treatment, rehabilitation, leisure, and entertainment for the elderly [11]. However, it is difficult to achieve the purpose of the elderly care institutions. It is urgent to improve the management team by industrialized, systematic, and efficient management. However, the current elderly care institutions hardly provide professional, systematic, and efficient care for the elderly. Therefore, it is extremely essential to improve the quality of managers and hence improve the quality of the elderly care service [12].

The quality and ability of the managers of the elderly care institutions are directly related to the professional level of the staff of the elderly care institutions, the quality of life of the elderly, and the operating efficiency of the elderly care institutions [13]. Therefore, it is necessary to carry out comprehensive training regularly for managers and medical staff. In order to meet the increasingly changing needs of elderly care services, basic and high-end special training should be provided, such as training on the knowledge of elderly care services, communication skills, management skills, professional attitude, life care skills, clinical care skills, and marketing knowledge. It is worth noting that the elderly care institutions combined with medical and health care have high requirements for the quality and ability of managers [5]. Young managers with the low education level and weak professional knowledge should be given priority training. Expanding the training scope mainly includes professional ethics, knowledge quality, ability quality, and psychological quality [14]. Among them, professional ethics is the primary foundation. Only those who are gentle, kind-hearted, responsible, and love the job of elderly care will devote themselves to the elderly care service. Therefore, some scholars have proposed that it is particularly important to strengthen the cultivation of professional ethics [15].

### 3.2. Improving the Salary to Enhance the Stability of the Manager's Team of Elderly Care Institutions Is Important

The results showed that 15% of the managers were not satisfied with the work state. 3.33% of the managers had a monthly income of less than ¥2000, more than half of the managers had a monthly salary of less than ¥3000, and only one manager had a salary of more than ¥5000. The salary is low, lower than the per capita disposable income of urban residents in the same year. The managers with the higher education level have more space for career growth, but the difference in the salary level is not significant. At present, the nurses in the elderly care institutions are mainly married women with old age. Their comprehensive quality and professional skills are relatively low. Meanwhile, they have a large workload and little social security [16]. It is difficult for elderly care institutions to attract professional staff involved because the young people are not willing to engage in elderly care services, and the salary provided is low.

Currently, the operation and financing methods of elderly care institutions are not scientific. Zhang Dan believed that a medical cost guarantee mechanism is unreasonable in China, and it is difficult for elderly care institutions to develop only supported by government funds [17]. Therefore, the government should increase funding to promote the development of elderly care institutions. However, some studies indicated that the way in which the government provided funds to elderly care institutions at one time was harmful to the sustainable development of elderly care services [4]. In addition, improving the financial support policy for the combination of medical and elderly care is essential. Governments should set up special funds and preferential policies for the combination of medical and health care institutions. Therefore, in order to stabilize and develop the management team of elderly care institutions, the government should increase investment to improve the salary and welfare of elderly care providers and eliminate dissatisfaction factors [18]. At the same time, it is very important to strengthen the vocational identity education of elderly care, enhance the intrinsic value and sense of achievement of elderly care, and hence attract highly educated professionals to join the management team. In addition, it is necessary to increase the community publicity to change the Chinese traditional concept of “raising children and preventing the aged” to encourage more young people to join the elderly care service.

### 3.3. Training the Professional Managers of the Elderly Care Institutions according to the National Guidelines for Combination of Medical and Elderly Health Care Is Urgent

In October 2019, the Ministry of Human Resources and Social Security and the Ministry of Civil Affairs issued and implemented the national vocational skills standard for nursing staff for the elderly care (2019 version) [19]. The occupation has five levels, including level 5 or junior, level 4 or intermediate, level 3 or senior, level 2 or technician, and level 1 or senior technician. This included the standards of dementia care, ability assessment, and quality management that were concerned by the society. The elderly care providers in the elderly care institutions must have corresponding certificates. The vocational skill training of the staff should adopt the unified standard and have examination. The corresponding vocational skill level certificate should be issued to the staff after passing the examination [20]. These have greatly broadened the professional field of the managers of the elderly care institutions, continuously selected and recruited excellent staff for the elderly care, and hence enriched and strengthened the elderly care management team. Meanwhile, the entry threshold and salary of the elderly care providers should be improved. Thus, it can improve the social status and professional skills of the elderly care providers. Only in this way can the team of elderly care providers be strengthened and the national elderly care service industry develop well. The major of elderly care of a higher vocational college in Central China has been recruiting students since 2018. There were 75 students from all over the country, with 9 boys. The college has provided workers of elderly care service for various institutions and communities. According to the research, only a small proportion of the elderly service and management students are still engaged in the industry five years after graduation. According to Herzberg's two factor theory, the quality of work state depends on the health care factors and incentive factors in work [21, 22]. Therefore, the simultaneous construction of care culture can optimize the ability of the team of elderly care and reduce the loss of elderly care providers [23, 24]. At the same time, all kinds of volunteers or social workers have been recruited to hold special lectures for managers of elderly care institutions regularly or provide medical support, psychological intervention, rehabilitation guidance, and other services for the elderly [25].

In fact, the combination of medical and health care could optimize the distribution of medical resources and satisfy the diversified needs of elderly care services [26]. It can effectively solve the problem of aging population and improve the health level of the elderly. Therefore, it is a feasible way for the development of elderly care institutional. The advantage of the combination of medical and health care is that the institutions can be equipped with medical facilities and medical staff, which can provide professional medical services for the elderly. However, there are still many specific problems in the elderly care service, such as the problem of the cooperation of various government departments and how to make a scientific and reasonable reimbursement ratio. Due to the imperfection service system of the combination of medical and elderly care, further investigation and research are needed on how to determine the access threshold of the corresponding elderly care institutions and whether the suggestions put forward by the authors are feasible for other regions.

## 4. Conclusions

In this study, most managers in elderly care institutions were middle-aged, with the low education level and years of management. By increasing financial input, formulating preferential policies, improving wages and welfare benefits, and reducing brain drain stabilize the management team of elderly care institutions. By focusing on the training to young managers with low education background and weak professional knowledge and expanding the scope of training, the comprehensive quality of elderly care managers could be improved. To further improve the comprehensive management quality of the elderly care institutions, the enrollment of colleges and universities should be expanded.

## Figures and Tables

**Figure 1:** Status of training level comparison across education level.

**Table 1:** Status of the managers of the elderly care institutions in a city in Central China (*n* = 60).

Variables	*n* (%)
Gender	
Women	40 (66.67)
Men	20 (33.33)

Types of qualifications	
None	6 (10.00)
Social workers	1 (1.67)
Geriatric nurses	44 (73.33)
Nurses	3 (5.00)
Doctors	1 (1.67)
Other professionals.	5 (8.33)

Exertion degree	
Exhausted	50 (83.33)
General	9 (15.00)
Easy	1 (1.67)

Household location	
Local countries	14 (23.33)
Changde City	42 (70.00)
Hunan province	4 (6.67)
Other provinces	0 (0.00)

Education level	
Under middle school	15 (25.00)
Middle school or high school	24 (40.00)
Technical college	16 (26.67)
University	5 (8.33)
Master's degree or above	0 (0.00)

Current income (¥)	
＜2000	2 (3.33)
2000∼3000	35 (58.33)
3000∼5000	22 (36.67)
>5000	1 (1.67)

Professional affection*∗*	
Very satisfied	28 (46.67)
Satisfied	23 (38.33)
Dissatisfied	9 (15.00)

Postadaptability	
Very adaptable	26 (43.33)
Adaptable	29 (48.33)
General	5 (8.33)
Uncomfortable	0 (0.00)
Very uncomfortable	0 (0.00)

Job mobility	
Yes	1 (1.67)
Not temporary	38 (63.33)
No	21 (35.00)
Daily sleep time	
＜4 hr	1 (1.67)
4∼6 hr	24 (40.00)
7∼8 hr	26 (43.33)
>8 hr	9 (15.00)

Expected income per month (¥)	
2000∼2999	1 (1.67)
3000∼3999	9 (15.00)
4000∼4999	27 (45.00)
5000∼5999	8 (13.33)
>6000	15 (25.00)

Training (MCQ)	
Never	3 (5.00)
In workplace	42 (70.00)
Province or city level	34 (56.67)
State level	7 (11.67)

Career growth space	
Little	12 (20.00)
A little bit	30 (50.00)
Large	18 (30.00)

Age (years old)	
＜30	3 (5.00)
31∼40	11 (18.33)
41∼50	27 (45.00)
51∼60	17 (28.33)
>60	2 (3.33)

Type of training expected (MCQ)	
Communication	39 (65.00)
Management and marketing	31 (51.67)
Medical care	30 (50.00)

Years of management	
＜2	22 (36.67)
3∼5	22 (36.67)
5∼10	7 (11.67)
>10	9 (15.00)

Career prospects	
Not good, disrespectful	2 (3.33)
Time needed to change	15 (25.00)
Common	6 (10.00)
Good	22 (36.67)
Very fulfilling	15 (25.00)

^*∗*^Professional affection included professional identity, sense of honor, job satisfaction, and empathy.

**Table 2:** Status of types of qualifications comparison across management years (*n* = 60%).

Management years	None	Social workers	Geriatric nurses	Nurses	Doctors	Other	Total
<2	6 (27.27)	0 (0.00)	12 (54.55)	3 (13.64)	0 (0.00)	1 (4.55)	22
3∼5	0 (0.00)	1 (4.55)	18 (81.82)	0 (0.00)	1 (4.55)	2 (9.09)	22
5∼10	0 (0.00)	0 (0.00)	5 (0.00)	0 (0.00)	0 (0.00)	2 (28.57)	7
>10	0 (0.00)	0 (0.00)	9 (0.00)	0 (0.00)	0 (0.00)	0 (0.00)	9

Fisher's exact test, *P*=0.0230.

**Table 3:** Status of education level comparison across age (*n* = 60%).

Age (years old)	Middle school	High school	Technical college graduate	University graduate	Master's degree or above	Total
<30	1 (33.33)	0 (0.00)	2 (66.67)	0 (0.00)	0 (0.00)	3
31∼40	0 (0.00)	5 (45.45)	4 (36.36)	2 (18.18)	0 (0.00)	11
41∼50	8 (29.63)	11 (40.74)	5 (18.52)	3 (11.11)	0 (0.00)	27
51∼60	6 (35.29)	8 (47.06)	3 (17.65)	0 (0.00)	0 (0.00)	17
>60	0 (0.00)	0 (0.00)	2 (100)	0 (0.00)	0 (0.00)	2

Fisher's exact test, *P*=0.0921.

**Table 4:** Status of career rising space comparison across education level (*n* = 60%).

Degree or certification	Little	A little bit	Large	Total
Under middle school	8 (53.33)	7 (46.67)	0 (0.00)	15
Middle or high school	2 (8.33)	11 (45.83)	11 (45.83)	24
Technical college	2 (12.5)	10 (62.5)	4 (25.00)	16
University	0 (0.00)	2 (40.00)	3 (60.00)	5
Master's degree or above	0 (0.00)	0 (0.00)	0 (0.00)	0

Fisher's exact test, *P*=0.0019.

**Table 5:** Status of income comparison across education level (*n* = 60%).

Degree or certification	<2000	2000∼3000	3000∼5000	>5000	Total
Under middle school	1 (6.67)	12 (80)	2 (13.33)	0 (0.00)	15
Middle or high school	1 (4.17)	12 (50.00)	11 (45.83)	0 (0.00)	24
Technical college	0 (0.00)	9 (56.25)	6 (37.5)	1 (6.25)	16
University	0 (0.00)	2 (40.00)	3 (60.00)	0 (0.00)	5
Master's degree or above	0 (0.00)	0 (0.00)	0 (0.00)	0 (0.00)	0

Fisher's exact test, *P*=0.2369.

## Data Availability

The data used to support the findings of this study are available from the corresponding author upon request.

## Additional Points

*Strengths and Limitations of This Study*. This is the first study exploring the situation of managers of elderly care institutions in a city in Central China under the national guidelines for the combination of medical and elderly health care and their future training system.

Managers play an essential role in the elderly care institutions as they provide explicit goals and explain how individual efforts contribute to improving the quality of elderly care service. Managers also offer their staff training and support to do job regarding medical and elderly care. Therefore, the perception and ability of managers may be the breakthrough for improving the quality of elderly care service. The limitations of this study are descriptive study with small sample size, not exploring in depth the correlation behind the results. Follow-up studies seeking the effects of the long-term training system for managers of elderly care institutions may be needed.
